RETRACTED

# Inhibition of YAP function overcomes BRAF inhibitor resistance in melanoma cancer stem cells

**DOI:** 10.18632/oncotarget.22628

**Published:** 2017-11-22

**Authors:** Matthew L. Fisher, Daniel Grun, Gautam Adhikary, Wen Xu, Richard L. Eckert

**Affiliations:** ^1^ Department of Biochemistry and Molecular Biology, University of Maryland School of Medicine, Baltimore, Maryland, 21201, USA; ^2^ Department of Dermatology, University of Maryland School of Medicine, Baltimore, Maryland, 21201, USA; ^3^ Department of Reproductive Biology, University of Maryland School of Medicine, Baltimore, Maryland, 21201, USA; ^4^ The Marlene and Stewart Greenebaum Comprehensive Cancer Center, University of Maryland School of Medicine, Baltimore, Maryland, 21201, USA

**Keywords:** melanoma, YAP and TAZ, cancer stem cell, BRAF inhibitor, drug resistance

## Abstract

Treating BRAF inhibitor-resistant melanoma is an important therapeutic goal. Thus, it is important to identify and target mechanisms of resistance to improve therapy. The YAP1 and TAZ proteins of the Hippo signaling pathway are important drivers of cancer cell survival, and are BRAF inhibitor resistant factors in melanoma. We examine the role of YAP1/TAZ in melanoma cancer stem cells (MCS cells). We demonstrate that YAP1, TAZ and TEAD (TEA domain transcription factor) levels are elevated in BRAF inhibitor resistant MCS cells and enhance cell survival, spheroid formation, matrigel invasion and tumor formation. Moreover, increased YAP1, TAZ and TEAD are associated with sustained ERK1/2 activity that is not suppressed by BRAF inhibitor. Xenograft studies show that treating BRAF inhibitor-resistant tumors with verteporfin, an agent that interferes with YAP1 function, reduces YAP1/TAZ level, restores BRAF inhibitor suppression of ERK1/2 signaling and reduces tumor growth. Verteporfin is highly effective as concentrations of verteporfin that do not impact tumor formation restore BRAF inhibitor suppression of tumor formation, suggesting that co-treatment with agents that inhibit YAP1 and BRAF(V600E) may be a viable therapy for cancer stem cell-derived BRAF inhibitor-resistant melanoma.

## INTRODUCTION

Nearly one-half of metastatic melanoma patients harbor a BRAFV600 mutation, the most common being BRAF(V600E) [1]. These constitutively-active mutants stimulate ERK1/2 and other signaling pathways to drive tumor cell survival [2, 3]. Vemurafenib (PLX4032) and dabrafenib are BRAF inhibitors (BRAFi) that target BRAFV600-mutant metastatic melanoma and have been shown to improve survival [4]. These agents are remarkably effective, but the majority of patients ultimately become resistant [4, 5]. Tumor cells utilize a number of strategies to circumvent these inhibitors, including activation of alternate survival pathways [3]. Hippo is an important signaling pathway that controls tissue and organ size [6] and is comprised of Mst1/2 kinases that phosphorylate LATS1/2 kinases which phosphorylate the nuclear adaptor factors, YAP1 and TAZ. In proliferating cells, YAP1 and TAZ localize to the nucleus where they interact with TEAD (TEA domain) transcription factors to drive cell proliferation and survival. In contrast, activation of LATS1/2 results in YAP1 and TAZ phosphorylation which causes these proteins to relocate to the cytoplasm where they are degraded [6, 7] leading to reduced proliferation. Hippo signaling is frequently reduced in tumors leading to enhanced nuclear YAP1/TAZ accumulation and activation of cell proliferation [6, 8]. In melanoma, reduced Hippo pathway signaling is associated with enhanced tumor formation and metastasis [9–11]. Recent reports [12, 13] identify YAP1/TAZ as BRAFi resistance factors in melanoma. These studies suggest that BRAFi treatment promotes remodeling of the cytoskeleton that promotes nuclear accumulation and activation of YAP1/TAZ [13]. This is consistent with the known activation of YAP1 in response to cytoskeletal changes [14]. An additional study suggests that YAP1 confers apoptosis resistance by increasing BCL-xL expression [12].

RETRACTED

In the present report, we extend these studies using melanoma cancer stem cells (MCS cells) and show that BRAFi resistant MCS cells display elevated YAP1, TAZ and TEAD levels, and that this is associated with enhanced spheroid formation, matrigel invasion and tumor formation, and that YAP1, TAZ or TEADs knockdown reduces these responses. Moreover, knockdown of individual TEAD proteins reduces matrigel invasion, but optimal suppression is observed following simultaneous knockdown of all four TEAD proteins. We further show that inhibition of YAP1 using verteporfin, an FDA approved drug [15] that inhibits YAP1 function [16–18], reduces YAP1/TAZ level and restores sensitivity to BRAFi. A striking finding is that treatment with low levels of verteporfin completely restores BRAFi suppression of tumor formation in BRAFi-resistant xenograft tumor models. This finding suggests that verteporfin, and related compounds, may be useful therapeutic agents in BRAFi-resistant melanoma.

## RESULTS

### YAP1 and TAZ are BRAFi resistance factors

PLX4032 is an important BRAF(V600E)-targeting drug used for the treatment of melanoma that is commercially available as vemurafenib [4]. PLX4032 is highly effective in the short-term, but the tumors eventually become resistant [4, 19]. As models to study PLX4032 drug resistance, we used BRAF(V600E)-positive/PLX4032-sensitive A375 cells and created PLX4032-resistant cells (e.g., A375-PLX-R) by selection in PLX4032 containing medium. Figure 1A shows that, unlike A375 cells, proliferation of A375-PLX-R cells is not suppressed by PLX4032. To understand the mechanism of resistance, we first confirmed that the YAP1 and TAZ transcription adaptor proteins, and the TEAD transcription factors, have a role in drug resistance [12, 13, 20–24]. Figure 1B shows that YAP1, TAZ and TEAD levels are increased in A375-PLX-R cells and that the increase in YAP1 level is associated with an increase in apparent YAP1 phosphorylation. Figure 1C shows that the YAP1 and TAZ increase is not due to a change in YAP1 or TAZ mRNA level. To confirm a biological role for these proteins, we performed knockdown and overexpression experiments. Figure 1D shows that treatment with PLX4032 or YAP1-siRNA reduces A375 cell proliferation, and that expression of constitutively active YAP1, YAP(S127A), reverses the PLX4032-dependent growth suppression. Moreover, we show that YAP1 knockdown reduces growth and restores A375-PLX-R cell response to PLX4032 (Figure 1D). TAZ also influences cell function. TAZ knockdown reduces A375 cell proliferation while TAZ overexpression partially reverses PLX4032-dependent growth suppression (Figure 1E). TAZ knockdown also partially restores sensitivity of A375-PLX-R cells to PLX4032 (Figure 1E). Figure 1F, 1G confirms the successful knockdown and overexpression of YAP1 and TAZ. These studies confirm previous studies [12, 13, 25] showing that YAP1 and TAZ are PLX4032 resistance factors.

RETRACTED

**Figure 1:** YAP1 and TAZ levels are elevated in A375-PLX-R cells and confer resistance to PLX4032 **(A)** A375 and A375-PLX-R cells were plated at equal density in growth medium and after overnight attachment were treated from 0 - 3 d with 0 or 1 μM PLX4032. **(B)** A375 and A375-PLX-R cells, growing in monolayer culture, were treated with 0 or 1 μM PLX4032 for 24 h and extracts were prepared to assay YAP1, TAZ and TEAD level. **(C)** Cells were grown in monolayer culture and extracts were prepared for qRT-PCR detection of YAP1 and TAZ mRNA. **(D, E)** A375 and A375-PLX-R cells were double-electroporated with 3 μg of Control-, YAP1- or TAZ-siRNA, or 2 μg of YAP(S127A), TAZ(S89A) or empty vector (EV), and after overnight attachment grown as monolayer cultures in the presence of 0 or 1 μM PLX4032. **(F, G)** Extracts were prepared from the cells described in panels D/E, at three days of treatment, and assayed by immunoblot to confirm YAP1 and TAZ knockdown and to demonstrate YAP(S127A) and TAZ(S89A) expression. The plotted values are mean ± SEM and asterisks indicate a significant reduction compared to control (n = 3, p < 0.005).

RETRACTED

### Role of YAP1 and TAZ in MCS cells

MCS cells can be selected by growth as spheroids and form rapidly growing, invasive and highly aggressive tumors as compared to non-stem melanoma cancer cells [26]. We therefore assayed the impact of PLX4032 treatment on MCS cell spheroids. Figure 2A, 2B shows that PLX4032 treatment suppresses A375 cell, but not A375-PLX-R cell, spheroid formation. Figure 2C shows that A375-PLX-R cell-derived MCS cells express elevated YAP1, TAZ and TEAD levels as compared to A375 cell derived MCS cells. In addition, YAP1-*P* formation is increased and TAZ-*P* formation reduced. These results are generally consistent with observations in monolayer culture (Figure 1). Subcellular distribution is reported to influence YAP1 and TAZ activity in some cell types and so we determined if PLX4032 treatment influences YAP1/TAZ subcellular distribution. As shown in Figure 2D, we did not observe a major change in YAP1 intracellular distribution in control versus PLX4032-treated A375 cells, suggesting that altered YAP1/TAZ subcellular distribution does not explain the response to PLX4032.

**Figure 2:** PLX4032 impact on A375 and A375-PLX-R cell spheroid formation and invasion **(A, B)** A375 and A375-PLX-R cells were plated in ultra-low attachment plates in spheroid medium, treated with the indicated doses of PLX4032, and spheroid number was monitored. **(C)** Spheroids were grown for 6 d in the presence of 0 or 1 μM PLX4032 prior to harvest, and lysates were prepared for detection of the indicated epitopes. **(D)** A375 cells were seeded on chamber slides, treated with 0 or 1 μM PLX4032 for 24 h, then fixed, permeabilized and incubated with primary antibodies specific for the indicated epitope and appropriate secondary antibody (C, control - indicates a staining control where sections were incubated with the secondary antibody alone). **(E)** A375 and A375-PLX-R cells were seeded atop a matrigel-coated membrane, in growth medium containing 0 or 1 μM PLX4032 for invasion assay. After 20 h, the membrane was removed, rinsed and fixed, and DAPI-stained nuclei were counted on the underside of the membrane. **(F, G)** A375 and A375-PLX-R cells were double-electroporated with 3 μg of Control-, YAP1- or TAZ-siRNA, or 2 μg of empty (EV), YAP(S127A) or TAZ(S89A) vector and plated atop a matrigel-coated membrane in growth medium containing 0 or 1 μM PLX4032. After 18 h, the membranes were fixed and stained with DAPI to visualize migrated cells. The values are mean ± SEM, n = 3. Asterisks indicate a significant reduction relative to control, p < 0.005.

We next measured PLX4032 impact on A375 and A375-PLX-R cell invasiveness using a matrigel invasion assay. MCS cells display enhanced invasion which is a measure of metastatic aggressiveness [26]. Figure 2E shows that A375-PLX-R cell invasion is enhanced by 50% compared to A375 cells, but that invasion is not suppressed by PLX4032 in either cell type. Figure 2F, 2G shows that although YAP1 or TAZ knockdown reduces invasion, PLX4032 treatment has no impact. These findings indicate that YAP1/TAZ knockdown does not sensitize the cells to PLX4032 with respect to matrigel invasion.

RETRACTED

The above findings show that YAP1 and TAZ antagonize PLX4032 suppression of proliferation and spheroid formation. To understand the molecular mechanism of this antagonism, we monitored signaling changes in A375 cells following expression of YAP(S127A) and TAZ(S89A) and challenge with PLX4032. YAP(S127A) and TAZ(S89A) are constitutively actives forms of these proteins. Consistent with previous reports, BRAFi treatment reduces A375 cell ERK1/2 activity (Figure 3A, 3B). Moreover, this is associated with reduced cyclin B and cyclin A, and increased p21^Cip1^ and p27 (Figure 3A, 3B). PLX4032 treatment also enhances apoptosis as measured by increased accumulation of cleaved PARP and reduced levels of procaspase 8 and 9. Consistent with a role for YAP1/TAZ in attenuating PLX4032 action, these changes are reversed by expression of constitutively-active forms of YAP1 (Figure 3A) or TAZ (Figure 3B). These findings are consistent with a previous report suggesting that YAP1 and TAZ antagonize BRAFi action by suppressing apoptosis [12]. In addition, ERK1/2 signaling is suppressed in response to PLX4032 in A375 cells, but YAP(S127A) or TAZ(S89A) expression restores and maintains ERK1/2 signaling that is not reduced by PLX4032 treatment (Figure 3A, 3B).

**Figure 3:** The role of YAP1, TAZ and TEADs **(A, B)** A375 cells were double-electroporated with empty vector (EV), YAP(S127A) or TAZ(S89A) encoding vector, plated and after attachment treated for 24 h with 0 or 1 μM PLX4032. Lysates were then collected for immunoblot. **(C)** A375 cells were electroporated with each of the indicated constructs and then plated for growth or invasion assays in the presence of 0 or 1 μM PLX4032. For the proliferation study, PLX4032 was added after cell attachment/recovery and cell number was determined at 3 d. For invasion assay, the membranes were fixed, and DAPI stained after 24 h to detect invading cells. The values are mean ± SEM, n = 4. **(D, E)** A375 or A375-PLX-R cells were double-electroporated with the indicated siRNA and permitted to recover before plating 25,000 cells atop a matrigel-coated membrane for invasion assay in the presence of 0 or 1 μM PLX4032. After 18 h, the membranes were fixed, and DAPI stained to detect invading cells. The values are mean ± SEM, n = 4. Asterisks indicate a significant reduction compared to control, p < 0.005. **(F)** A375 and A375-PLX-R cells were double-electroporated with pooled siRNA against TEAD1, 2, 3, and 4 (0.75 μg each). At 24 h post-electroporation, the cells were treated with 1 μM PLX4032 for 24 hours and lysates were collected for immunoblot.

RETRACTED

### Role of TEAD transcription factors in MCS cells

YAP1 interacts in the nucleus with TEAD transcription factors to regulate gene expression leading to enhanced cell proliferation and survival [6, 16]. Since YAP1 can also interact with other targets [27], we determined whether YAP1/TEAD interaction is required for PLX4032 resistance. Figure 3C shows that YAP(S127A) expression can reverse PLX4032 suppression of A375 cell proliferation. We then monitored the ability of YAP(S127A) mutants, which cannot interact with selected cellular proteins, to replicate this response. YAP(S127A)(S94A) is a TEAD interaction domain mutant that is unable to interact with TEAD factors. YAP(S127A)(WW1), YAP(S127A)(WW2) and YAP(S127A)(WW1/WW2) have mutations in key tryptophan resides in the WW domains and cannot interact with WW domain binding proteins. YAP(S127A)(Dbl) is a double mutant combining the S94A and WW domain mutations, and YAP(S127A)(PDZbm) has a c-terminal 5 amino acid truncation that removes the PDZ binding domain [8]. We show that all of these constructs are able to restore cell proliferation in PLX4032-treated A375 cells, except for YAP(S127A)(S94A) and YAP(S127A)(Dbl). Both of these mutants encode the S94A mutation in the TEAD interaction domain which inactivates interaction with TEAD factors (Figure 3C, upper panel). This indicates that YAP1 antagonism of PLX4032-dependent growth suppression requires YAP1 interaction with TEAD factors. We next measured the impact of each mutant and PLX4032 treatment on A375 cell matrigel invasion. Figure 3C (lower panel) tests the requirement for YAP1/TEAD interaction in this context. This data confirms, as shown in Figure 2F, that YAP1 stimulates and PLX4032 does not regulate invasion. It also shows that all YAP(S127A) forms increase A375 cell matrigel invasion, except for the YAP(S127A)S94A and YAP(S127A)Dbl mutants that do not interact with TEAD factors.

We next examined the impact of TEAD factor knockdown on invasion in PLX4032 sensitive and resistant cells. PLX4032 resistant cells more efficiently invade matrigel as compared to PLX4032 sensitive cells (compare control group values in Figure 3D and 3E). Moreover, loss of individual TEAD proteins reduces invasion, and simultaneous loss of all TEAD factors results in the greatest reduction (Figure 3D, 3E). TEAD loss reduces PLX4032-resistant cell invasion (Figure 3E) to the level observed in untreated PLX4032-sensitive A375 cells (Figure 3D); however, PLX4032 treatment does not impact invasion (Figure 3D, 3E). We next examined the impact of PLX4032 on signaling in TEAD intact and knockdown A375 and A375-PLX-R cells. ERK1/2 phosphorylation is particularly interesting in that it is reduced in PLX4032-treated A375 cells in the presence or absence of TEADs. In contrast, ERK1/2 activity is only reduced in A375-PLX-R cells following TEAD knockdown and PLX4032 treatment (Figure 3F). In contrast, TEAD knockdown does not appreciably alter YAP1, YAP1-*P*, TAZ or TAZ-*P* levels in either cell line, and p21^Cip1^ levels are increased by PLX4032 treatment or TEAD knockdown (Figure 3F).

RETRACTED

### Pharmacologic inhibition of YAP1 and BRAF(V600E) on MCS cell survival

Identification of agents that suppress survival of PLX4032-resistant cells, or re-sensitize these cells to PLX4032, is an important goal. The experiments in Figure 1D suggest that interfering with YAP1 function may achieve this objective. YAP1 interacts with TEAD transcription factors to drive gene expression [6, 28] and a small molecular inhibitor called verteporfin has been reported to disrupt YAP1/TEAD interaction by binding to YAP1 and altering its structure [6, 16]. We therefore examined the impact of verteporfin treatment on spheroid formation and matrigel invasion in PLX4032 sensitive and resistant MCS cells. Figure 4A, 4B shows that verteporfin treatment suppresses A375 and A375-PLX-R spheroid formation by 50% at verteporfin concentrations as low at 0.1–0.25 μM and that spheroid formation is nearly completely inhibited at higher verteporfin concentrations. We also studied the effect of verteporfin on pre-formed spheroids. In this assay, spheroids are permitted to form for 8 d and then treated with verteporfin. We observe that 20 μM verteporfin treatment reduces spheroid number/integrity (Figure 4C) by 30 - 50% after a 3 d treatment. Prolonged treatment results in complete destruction of the spheroids (not shown). We next examined the impact of verteporfin on ability to invade matrigel. Figure 4D, 4E shows that matrigel invasion is 50% suppressed at concentrations of 0.5 - 1 μM verteporfin and that suppression is nearly complete at higher concentrations.

**Figure 4:** Verteporfin suppression of spheroid formation and invasion is associated with reduced YAP1/TAZ level **(A, B)** A375 or A375-PLX-R cells (40,000) were seeded in ultra-low attachment plates in spheroid medium, treated with verteporfin, and spheroid number was recorded and images derived at the indicated times. **(C)** A375 and A375-PLX-R cells were seeded in ultra-low attachment plates in spheroid medium and grown as spheroids for 8 d. Verteporfin treatment was initiated and spheroid number counted after 3 d. **(D, E)** A375 or A375-PLX-R cells were seeded for invasion assay on a matrigel-coated membrane in growth medium containing 0 - 20 μM verteporfin. After 18 h the membrane was removed and DAPI stained to visualize invading cells on the underside of the membrane. **(F)** A375 and A375-PLX-R cells were treated for 1 μM verteporfin for 48 h and mRNA extracts were prepared for assay of YAP1 and TAZ mRNA by qRT-PCR. **(G, H)** A375 and A375-PLX-R cells were plated for spheroid formation followed by addition of 1 μM verteporfin and incubation for 6 d prior to preparation of extracts for immunoblot detection of YAP1, TAZ and pan-TEAD. **(I)** A375 monolayer cells were pre-treated with 1 μM lactacystin for 1 h followed by addition of 5 μM verteporfin. Lysates were collected after 24 h for immunoblot. The values are mean ± SEM, n = 3 and the asterisks indicate a significant reduction relative to control, p < 0.005.

RETRACTED

To understand the mechanism of verteporfin action, we treated monolayer A375 and A375-PLX-R cells with 1 μM verteporfin for 24 h and then monitored the impact on YAP1/TAZ mRNA and protein level. Verteporfin treatment does not impact the level of YAP1 or TAZ mRNA (Figure 4F), but does reduce YAP1 and TAZ protein level (Figure 4G). As shown in Figure 4H, verteporfin treatment also reduces TEAD transcription factor level. The proteasome is known to regulate YAP1/TAZ level [29, 30] and so we examined whether the proteasome is responsible for the observed reductions. Figure 4I shows the verteporfin-dependent reduction in YAP1, TAZ and TEAD level is not reversed by the proteasome inhibitor, lactacystin.

We next assayed whether verteporfin treatment can restore PLX4032 sensitivity in resistant cells. A375-PLX-R cells were plated in spheroid growth conditions and treated with 0–1 μM PLX4032 in the presence of 0 or 1 μM verteporfin and spheroid formation was monitored. Figure 5A confirms that treatment with 0–1 μM PLX4032 does not suppress A375-PLX-R spheroid formation, but that co-treatment with 0.1 μM verteporfin restores PLX4032 suppression of spheroid number.

**Figure 5:** Verteporfin impact on other PLX4032-resistant melanoma cancer cells **(A)** Verteporfin restores sensitivity to PLX4032. A375-PLX-R cells were plated for spheroid formation assay in the presence of the indicated level of PLX4032 and verteporfin which was added the morning after plating. Spheroids were counted at 2, 6 and 10 days. **(B)** PLX4032-resistant cell lines were harvested, and 40,000 cells were plated in spheroid growth conditions followed by treatment with 0 or 1 μM PLX4032 and counting of spheroid number after 8 d. **(C)** PLX4032-resistant cell lines were harvested, and 25,000 cells were plated on a matrigel-coated membrane for invasion assay in the presence of 0 or 1 μM PLX4032. After 18 h, the membranes were removed, fixed, and DAPI stained to detect invading cells on the membrane. **(D)** The indicated melanoma cancer cell lines, maintained in growth medium, were treated for 24 h with 0 or 1 μM PLX4032 and extracts were prepared for immunoblot detection of the indicated proteins. **(E)** PLX4032-resistant cell lines were harvested, and 40,000 cells were plated in spheroid growth conditions followed by treatment with 0 or 5 μM verteporfin and counting of spheroids after 8 d. **(F)** PLX4032-resistant cell lines were harvested, and 25,000 cells were plated on a matrigel-coated membrane for invasion assay in the presence of 0 or 5 μM verteporfin. After 18 h, the membranes were removed, fixed, and DAPI stained to detect cells that migrated through the matrigel. **(G)** SK-MEL-28 cells were double-electroporated with 3 μg of YAP(S127A), TAZ(S89A) or empty (EV) vector and then grown as monolayer cultures in the presence of 0 or 1 μM PLX4032. Cells were counted at the indicated times. **(H)** PLX4032 resistant A375-PLX-R cells were plated in 35 mm dishes. After 24 h, treatment was initiated with 0 or 1 μM SCH772984 and cells were counted at the indicated times. **(I)** PLX4032 resistant cells were plated in 35 mm dishes. After 24 h, treatment was initiated with 0 or 1 μM SCH772984 and cells were counted at 3 d. The values are mean ± SEM and asterisks indicate a significant difference compared to control, n = 3, p < 0.005.

RETRACTED

### Verteporfin suppresses survival of other PLX4032-resistant cell lines

We next examined the impact of verteporfin on additional PLX4032 resistant melanoma cancer cell lines. SK-MEL-5, SK-MEL-28 and WM3248 cells were selected for PLX4032 resistance by continuous growth in medium containing 1 μM PLX4032. Figure 5B, 5C confirms that PLX4032 treatment does not reduce spheroid formation or matrigel invasion in these lines. Consistent with our findings in A375 and A375-PLX-R cells, YAP1, TAZ and TEAD levels are markedly increased in the resistant lines (Figure 5D), a finding that is consistent with the hypothesis that these transcriptional regulators can contribute to PLX4032 resistance. We next monitored the effect of verteporfin on biological endpoints. Figure 5E, 5F shows that verteporfin treatment reduces spheroid formation and matrigel invasion. To determine whether YAP1 and TAZ can antagonize PLX4032 action, we expressed constitutively active YAP1 and TAZ in wild-type SK-MEL-28 cells and monitored impact on cell proliferation. Figure 5G shows that forced expression of YAP(S127A) or TAZ(S89A) partially reverses PLX4032 suppression of cell growth.

### PLX4032 resistant cell response to ERK inhibitor

Our findings suggest that YAP1/TAZ and TEADs foster melanoma cancer cell survival by maintaining ERK1/2 signaling as a mechanism to circumvent BRAF(V600E) inhibition (Figure 3A, 3B, 3F). This predicts that the BRAFi-resistant cells should remain sensitive to ERK1/2 inhibitors. To assess the role of ERK1/2 we treated PLX4032 resistant cells with SCH772984, a specific inhibitor of ERK1/2 [31], and monitored the impact on cell proliferation. SCH772984 treatment produces a time-dependent reduction in A375-PLX-R cells number (Figure 5H) and also reduces proliferation of SKMEL5-PLX-R, SKMEL28-PLX-R and WM3248-PLX-R cells (Figure 5I).

### Impact of verteporfin and BRAFi co-treatment on tumor formation

We next monitored the impact of verteporfin on melanoma cell tumor formation. We selected MCS cells as these cells display markedly enhanced malignant potential [26]. A375-PLX-R derived MCS cells form large tumors compared to A375 MCS cells (Figure 6A), and PLX4032 suppresses growth of A375 but not A375-PLX-R spheroid cell-derived tumors (Figure 6B). Moreover, consistent with the cell culture findings, the A375-PLX-R spheroid cell-derived tumors express elevated levels of YAP1, TAZ and TEADs as compared to A375 spheroid cell-derived tumors (Figure 6C). In addition, ERK1/2-*P*, cyclins A and B, and CDK4 levels are elevated in A375-PLX-R spheroid cell-derived tumors (Figure 6C). p21^Cip1^ level is selectively slightly elevated in PLX4032-treated A375 spheroid cell-derived tumors (Figure 6C), a finding that is consistent with their sensitivity to PLX4032 growth inhibition. The increase in YAP1, TAZ and TEADs in PLX4032 resistant tumor-derived MCS cells reflects the changes observed in cultured PLX4032-resistant cells (Figure 2C), and indicates that elevated levels of YAP1, TAZ and TEAD factors are retained during growth in PLX4032 resistant tumors. We next assessed the impact of inhibiting YAP1 function on tumor formation. Figure 6D and E shows that verteporfin treatment suppresses YAP1 and TAZ level and that this is associated with reduced tumor size.

**Figure 6:** Verteporfin impact on tumor formation **(A)** Spheroid culture-derived A375 and A375-PLX-R cells were injected at 0.1 million per each front flank and tumor formation was monitored for 4 wks. The asterisk indicates a significant increase in the A375-PLX-R spheroid tumor size compared to the A375 spheroid group, p < 0.005 **(B)** Spheroid culture-derived A375 and A375-PLX-R cells were injected at 0.1 million cells per each front flank followed by PLX4032 treatment and monitoring of tumor growth for 4 wks. The asterisk indicates a significant reduction in tumor size compared to control group, p < 0.005. **(C)** Extracts were prepared from A375 and A375-PLX-R tumors (4 wks) from panel B for immunoblot detection of the indicated epitopes. **(D, E)** A375-PLX-R cells were injected at 0.1 million cells/each front flank and verteporfin treatment was initiated. Extracts were prepared to monitor YAP1 and TAZ levels in control and verteporfin-treated tumors. The asterisk indicates a significant reduction compared to the control group, p < 0.005. **(F, G)** Spheroid culture-derived A375 and A375-PLX-R cells were grown as tumors for 4 wk with the indicated drug treatment. The tumors were removed and single cell suspensions prepared for matrigel invasion assay. Cells were plated at 25,000 cells per well atop a Matrigel layer in a Millicell chamber in the absence of drug for invasion assay. The labels indicate the drug treatment administered during tumor growth. After 18 h, the membrane was recovered to count migrated cells [38]. The asterisks indicate a significant increase in invasion compared to the A375 spheroid tumor-derived cells, and the double asterisks indicate a reduction in invasion compare to the A375-PLX-R spheroid tumor-derived cells, p < 0.005.

RETRACTED

To measure whether verteporfin treatment influences the cancer stem cell status in the tumor, we harvested the tumor cells and monitored efficiency of matrigel invasion in the absence of drug treatment. Figure 6F shows that the tumor-derived A375-PLX-R cells invade matrigel nearly three times as efficiently as tumor-derived A375 cells, and that *in vivo* PLX4032 treatment does not suppress matrigel invasion of sensitive or resistant cells (Figure 6F). In contrast, verteporfin treatment of tumors reduces tumor formation and yields a cell population with reduced matrigel invasion (Figure 6G).

### Verteporfin treatment restores tumor response to BRAFi

We surmised that inhibition of YAP1 function may restore PLX4032 suppression of tumor formation. To test this we measured the impact of treatment with 20 mg/kg PLX4032 in the presence of 0 - 100 mg/kg verteporfin on tumor formation by spheroid-derived A375-PLX-R cells. Figure 7A, 7B shows that in the absence of verteporfin, PLX4032 does not suppress A375-PLX-R tumor formation. However, verteporfin treatment produces a dose-dependent reduction in tumor size. The key observation is that treatment with a low concentration of verteporfin (10 mg/kg), that does not suppress tumor formation, restores PLX4032-dependent suppression of tumor formation. An examination of the biochemical status of the 10 mg/kg verteporfin plus 20 mg/kg PLX4032-treated tumors reveals a reduction in YAP1, YAP1-*P*, TAZ and TEAD levels (Figure 7C). In addition, in the presence of verteporfin, PLX4032 treatment reduces ERK1/2-*P* level. These findings show that treatment with low levels of verteporfin, that do not impact tumor formation, can re-sensitize tumors to PLX4032.

RETRACTED

**Figure 7:** Verteporfin restores PLX4032 suppression of ERK1/2 signaling and tumor formation **(A, B)** Spheroid-derived A375-PLX-R cells were injected in each front flank followed by verteporfin and PLX4032 treatment and monitoring of tumor growth for 4 wks. The values are mean ± SEM. The asterisks indicate a significant reduction compared to verteporfin alone, p < 0.001. **(C)** Tumor extracts were from tumor treated with prepared for detection of signaling proteins. For all figure panels, the asterisks indicate a significant increase compared to control. The values are mean ± SEM, n = 3, p < 0.005.

## DISCUSSION

### YAP1 and TAZ are BRAFi resistance factors

Nearly one-half of all patients with metastatic melanoma harbor a BRAF(V600) mutation, the most common being BRAF(V600E) [1]. These mutants are constitutively active monomers which hyperactivate ERK signaling [2, 3]. Vemurafenib (PLX4032) and dabrafenib are inhibitors that target BRAF(V600E)-positive melanoma. Although these drugs improve progression-free survival by ten months and overall survival by twelve months [4], most patients ultimately become resistant [4, 5]. Thus, it is important to identify BRAFi resistance mechanisms that can be targeted to restore BRAFi activity [3].

Hippo signaling is an important evolutionarily-conserved signaling pathway that controls tissue and organ size during development [6]. Contact inhibition of cell proliferation is associated with activation of the Hippo signaling kinases, Mst1/2 and LATS1/2, leading to YAP1 and TAZ phosphorylation and degradation [7]. In contrast, LATS1 activity is reduced in proliferating cells leading to YAP1/TAZ accumulation in the nucleus and interaction with TEAD transcription factors to drive transcription of pro-growth/pro-survival genes [6]. The YAP1/TAZ transcription adaptor proteins and TEAD transcription factors are also important regulators in cancer cells, as Hippo activity is often reduced in tumors leading to increased nuclear accumulation of non-phosphorylated YAP1 and TAZ, and activation of proliferation-associated transcription and cell survival [6, 8]. YAP1, TAZ and TEAD can also mediate drug resistance [12, 23, 24]. In melanoma, reduced Hippo signaling activity and increased YAP1 function is associated with enhanced melanoma cell survival [9–12].

RETRACTED

### YAP1 and BRAFi impact on MCS cell spheroid formation and matrigel invasion

Our present studies expand these studies by examining the role of YAP1/TAZ/TEAD in MCS cells and the impact of BRAFi and verteporfin treatment. We show that BRAFi and YAP1/TAZ/TEAD regulate responses that are enhanced in MCS cells including cell proliferation, spheroid formation and matrigel invasion. Selection with PLX4032 leads to BRAFi resistance and this is associated with a marked increase in YAP1, TAZ and TEAD levels and enhanced spheroid formation potential. This is biologically meaningful, as YAP1 or TAZ knockdown in BRAFi-resistant MCS cells, restores BRAFi sensitivity, and forced expression of constitutively active YAP1 or TAZ confers BRAFi resistance on sensitive cells. This role for YAP1 and TAZ was observed in PLX4032 resistant cell lines derived from A375, SK-MEL-5, SK-MEL-28 and WM3248 cells. These findings confirm that BRAFi resistance in MCS cells is associated with enhanced expression of YAP1, TAZ and TEADs, a finding previously reported in non-stem melanoma cancer cells [9–12].

Matrigel invasion is a measure of MCS cell metastatic potential. Our studies reveal potentially important and unexpected features regarding melanoma cancer cell invasion, the role of YAP1/TAZ in this process, and the response to PLX4032 treatment. YAP1, TAZ and TEAD knockdown reduces MCS cell invasion and YAP1 or TAZ overexpression increases invasion, showing that YAP1, TAZ and TEADs play a key role in regulating this process. These findings are consistent with a study showing that YAP1 is required for metastasis of tail vein-injected melanoma cells [11]. In contrast, it is interesting that although PLX4032 suppresses MCS cell proliferation and spheroid formation, it does not suppress invasion in BRAFi sensitive or resistant MCS cells. This interesting finding indicates that PLX4032 does not suppress all biological responses associated with the MCS cell phenotype nor does it oppose all YAP1/TAZ/TEAD-stimulated biological responses. These findings have important implications for therapy, and suggest that the YAP1/BRAFi interplay may be more complicated than previously appreciated.

### YAP1/TAZ and BRAFi impact on MCS cell signaling

BRAF(V600E) drives melanoma cell survival by activating ERK1/2 signaling [32]. We therefore studied the impact of PLX4032 on ERK1/2 level and phosphorylation. In inhibitor sensitive cells, PLX4032 suppresses ERK1/2 phosphorylation. In contrast, PLX4032 does not suppress ERK1/2 signaling in BRAFi-resistant cells. Moreover PLX4032 does not suppress ERK1/2 activity when constitutively-active YAP1 or TAZ are expressed in PLX4032-sensitive cells. These findings are consistent with previous reports [12, 33], and suggest that YAP1 and TAZ antagonize BRAFi action by maintaining ERK1/2 activity. If ERK1/2 is the key mediator, we would expect that ERK1/2 inhibitors should reduce BRAF-resistant cell survival and proliferation. In fact, treatment with an ERK1/2 specific inhibitor, SCH772984, suppresses survival of BRAFi resistant cells, suggesting that ERK1/2 activity is a key nexus that mediates YAP1/TAZ-associated resistance. Additional studies will be required to understand this role. PLX4032 treatment also reduces cyclin A and cyclin B level and increases p21^Cip1^ and p27, findings that are consistent with BRAFi suppression of cell proliferation. In addition, PLX4032 treatment increases apoptosis, as measured by increased PARP cleavage and reduced procaspase level. These responses are reversed by expression of constitutively-active YAP1 or TAZ, consistent with the idea that BRAFi suppresses cell growth and enhances cell death, and YAP1/TAZ antagonize these actions [12, 25].

RETRACTED

### TEAD transcription factors

The four TEAD transcription factors (TEAD1/2/3/4) are major downstream targets of YAP1 and TAZ [34–37] and the observed increase in TEAD factor level in PLX4032 resistant cells is consistent with a role in BRAFi resistance. However, YAP1 and TAZ can interact with targets other than TEAD factors to guide responses [27] and so we used genetic and knockdown approaches to confirm that TEAD factors mediate the YAP1/TAZ antagonism of PLX4032 action. We show that constitutively-active YAP1 reverses PLX4032 suppression of cell proliferation, and mutants of constitutively-active YAP1 that cannot interact with TEAD factors lack this ability, suggesting that YAP1/TEAD interaction is required for BRAFi resistance. In addition, TEAD knockdown or treatment with BRAFi produces similar changes in signaling. For example, TEAD knockdown restores the ability of PLX4032 to reduce ERK1/2 activity. In addition, we assessed the role of TEAD1, 2, 3 and 4 in a matrigel invasion assay. Knockdown of individual TEAD factors resulted in a similar reduction in MCS cell matrigel invasion, and maximal suppression was observed in response to simultaneous knockdown of all four isoforms. This suggests that all of the TEAD factors have biological activity. Taken together, these findings suggest that TEAD factors are the likely downstream targets of YAP1/TAZ in MCS cells, and that YAP1/TAZ and TEAD factor interaction is required for MCS cell survival and BRAFi resistance.

RETRACTED

### Verteporfin treatment restores sensitivity of MCS cells to PLX4032

One of the most interesting aspects of this report are the tumor findings. Verteporfin is a small aromatic heterocyclic molecule that disrupts YAP1/TEAD interaction [16, 35], and is an FDA drug approved for photodynamic therapy of neovascular macular degeneration that is marketed as Visudyne by Novartis [15]. We show that PLX4032 resistant MCS cells form large and highly aggressive tumors compared to non-PLX4032 resistant cells. We selected the BRAFi-resistant MCS cells for tumor studies, since they are the most aggressive cells with respect to tumor formation. We show that treatment with verteporfin reduces tumor formation and YAP1, TAZ and TEAD levels. The ability of verteporfin to markedly suppress YAP1 and TAZ levels in cultured MCS cells suggested that it may be effective in restoration of BRAFi sensitivity in tumors. An important finding is that verteporfin reduces tumor growth and that this is associated with reduced YAP1/TAZ level. However, the most remarkable observation is that treatment with a concentration of verteporfin that does not suppress tumor formation restores PLX4032 suppression of tumor formation. A remarkable (80%) suppression of tumor size is observed in mice treated with the combination, and this was associated with PLX4032 suppression of ERK1/2 signaling in the verteporfin co-treated tumors. This combination of agents was well tolerated by the mice and suggests that verteporfin, or a related agent, may be useful in restore BRAFi action in human patients.

## MATERIALS AND METHODS

### Antibodies and reagents

Sodium pyruvate (11360-070), Dulbecco's Modified Eagle's Medium (DMEM) (11960-077), 0.25% trypsin-EDTA (25200-056) and L-Glutamine (25030-164) were purchased from Gibco (Grand Island, NY, USA). Heat inactivated fetal calf serum (FCS, F4135), anti-β-actin (A5441) and lactacystin (L6785) were purchased from Sigma (St. Louis, MO, USA). Cell lysis Buffer (9803) and antibodies for ERK1/2 (9102), ERK1/2-*P* (9101), YAP1 (4912), YAP1-*P* (13008), TAZ (4883) pan-TEAD (13295), p21^Cip1^ (2947), cleaved PARP (9541), caspase-8 (9746) and caspase-9 (9502) were from Cell Signaling Technologies (Danvers, MA, USA). Antibodies to cyclin A (SC-751), cyclin B (SC-245), p27 (SC-1641) and TAZ-*P* (SC-17610-R) were purchased from Santa Cruz (Dallas, TX, USA). YAP1 (52771) antibody for immunofluorescence was purchased from Abcam (Cambridge, MA, USA). YAP1-siRNA (S102662954, S104438651, S104438644, S104438637) were purchased from Qiagen (Valencia, CA, USA). Control- (37007) and TAZ-siRNA (36568) were purchased from Santa Cruz. TEAD1 (M-012603-01-0005), TEAD2 (M-012611-00-0005), TEAD3 (M-012604-01-0005) and TEAD4-siRNA (M-019570-03-0005) were purchased from Dharmacon. YAP(S127A) (27370) and TAZ(S89A) (32840) plasmids were obtained from Addgene (Cambridge, MA, USA). PLX4032 (RG7204) was purchased from APExBIO (Houston TX, USA). Peroxidase-conjugated anti-mouse IgG (NXA931) and anti-rabbit IgG (NA934V) were obtained from GE healthcare (Buckinghamshire, UK). Alexaflour 555 (A21424) and Alexaflour 488 (A11034) were purchased from Invitrogen. DAPI (D9542) was purchased from Sigma. Paraformaldehyde (15713) was purchased from Electron Microscopy Sciences (Hatfield, PA, USA). Matrigel (354234) and BD Biocoat cell inserts (353097) were purchased from BD Biosciences. Verteporfin (5305) was from Tocris Bioscience (Bristol, UK). Lab-Tek II Chamber Slides (154526) were from Nunc (Rochester, NY, USA). A375, SK-MEL-5, SK-MEL-28 and WM3248 cells, which harbor the BRAF(V600E) mutation, were kindly provided by Dr. David Kaetzel (Biochemistry and Molecular Biology, University of Maryland School of Medicine). YAP1 mutant plasmids were kindly provided by John Lamar/Richard Hynes [8]. These include YAP(S127A), YAP(S127A)(S94A), YAP(S127A)(WW1), YAP(S127A)(WW2), YAP(S127A)(WW1/WW2), YAP(S127A)(Dbl) and YAP(S127A)(PDZbm) [8]. The ERK1/2 inhibitor, SCH772984, was obtained from Selleckchem (Houston, TX, S7101). Data analysis used the student's t-test and values are presented as mean ± SEM.

RETRACTED

### Immunoblot and immuonstaining

Equivalent amounts of protein were electrophoresed on denaturing and reducing 10% polyacrylamide gels and transferred to nitrocellulose membrane. The membrane was blocked by 5% nonfat dry milk for one hour and incubated with 1:1000 primary antibody in 5% nonfat dry milk. Blots were rinsed in TBS-T and then incubated with secondary antibodies (1:5000) for 2 h. Secondary antibody binding was visualized using ECL Prime (Amersham) chemiluminescence detection technology. For immunostaining, cells were harvested, suspended in growth medium, and plated in LAB-TEK II Chamber Slide System. After 24 h, the cells were fixed with 4% paraformaldehyde at room temperature for 15 min, washed three times with phosphate-buffered saline, immersed in 0.1% Triton X-100 for 15 min, washed with phosphate-buffered saline, and blocked for 1 h with phosphate-buffered saline containing 7.5% fetal calf serum. Primary antibodies were added and the slides incubated overnight at 4°C. Cells were then washed three times with phosphate-buffered saline and incubated 1 h with the appropriate Alexa Flour fluorescence probe-conjugated secondary antibody. After additional washing, the cells were stained with DAPI for 10 min prior to imaging.

RETRACTED

### Spheroid formation assay

Cancer cells were maintained under attached conditions in growth media containing DMEM (Invitrogen, Frederick, MD, USA) supplemented with 4.5 mg/ml D-glucose, 2 mM L-glutamine, 1 mM sodium pyruvate, and 5% fetal calf serum. For spheroid culture, monolayer cultures were dissociated with 0.25% trypsin and the cells were collected by centrifugation, and resuspended in spheroid media, consisting of DMEM/F12 (1:1) (DMT-10-090-CV, Mediatech INC, Manassa, VA, USA) containing 2% B27 serum-free supplement (17504-044, Invitrogen, Frederick, MD, USA) 20 ng/ml EGF (E4269, Sigma, St. Louis, USA), 0.4% bovine serum albumin (B4287, Sigma) and 4 μg/ml insulin (19278 Sigma, St. Louis, MO, USA) and plated at 40,000 cells per 9.6 cm^2^ well in six well ultra-low attachment Costar cluster dishes (4371, Corning, Tewksbury, MA, USA). Parallel cultures were plated in spheroid media on conventional plastic dishes for growth as monolayer cultures.

### Electroporation of nucleic acids

Cancer cells (150,000) were plated on 60 mm plates in growth medium. After 24 h, when approximately 50% confluent, the cells were collected using 0.25% trypsin, centrifuged at 200 x g, washed with sterile PBS (pH 7.5), suspended in 100 μl of nucleofection reagent R VCA-1001 (Walkersville, MD, USA) and electroporated with plasmids or siRNA. The cell suspension, containing either 3 μg of siRNA or 2 μg of plasmid DNA was gently mixed and electroporated using the X-001 setting on the AMAXA Electroporator. Immediately after electroporation, pre-warmed media was added and the suspension was transferred to a 60 mm cell culture plate and a final volume of 4 ml of media. Cells were electroporated a second time, following the same protocol, 72 h after the initial electroporation.

### Invasion assay

Matrigel (BD Biolabs) was diluted in 0.01 M Tris-HCL/0.7% NaCl, filter sterilized and 0.1 ml was used to cover the membrane in BD BioCoat cell inserts (#353097, 8 μm pores, 24 well format, membrane growth area = 0.33 cm^2^). Cells 25,000/well were plated in 100 μl of growth media containing 1% FCS atop the Matrigel. Growth media containing 10% FCS was added to the lower well and cells were incubated overnight at 37 C. The following day, excess cells from the top side of the membrane were removed with a cotton swab, and the membrane was rinsed in phosphate-buffered saline, fixed with 4% paraformaldehyde for 10 minutes, washed and stained in 1 μg/ml DAPI for 10 minutes to visualize the cells. The underside of the membrane was photographed with an inverted fluorescent microscope to count the number of cells that had migrated through the Matrigel layer [38].

### PLX4032 resistant lines

A375, SK-MEL-5 and SK-MEL-28 cell lines were maintained in DMEM growth medium containing 10% FCS, 2 mM L-glutamine and 1 mM sodium pyruvate. The WM3248 cells were maintained in MCDB153:L15 (4:1) growth medium containing 2% FCS, 5 μg/ml insulin and 1.68 mM CaCl_2_. To create PLX4032-resistant cells, A375, SK-MEL-5, SK-MEL-28 and WM3248 cells were treated with 1 μM PLX4032 in monolayer culture in growth medium for several weeks. The surviving cells were then expanded and cultured in increasing doses of PLX4032 up to 4 μM. The resulting PLX4032-resistant cells, designated PLX4032-resistant (e.g., A375-PLX-R) were routinely maintained in the presence of 1 μM PLX4032.

RETRACTED

### Tumor xenograft assays

Cells were grown for ten days as spheroids and a single cell suspension, prepared by trypsin digestion, was resuspended in phosphate buffered saline containing 30% Matrigel and 100 μl containing 0.1 million cells were injected subcutaneously at the two front flanks of NOD/*scid*/IL2 receptor gamma-knockout mice (NSG mice) using a 26.5 gauge needle. PLX4032 was dissolved in phosphate-buffered saline containing 10% DMSO and delivered at 20 mg/kg by oral gavage in 100 μl three times per week (M/W/F). Verteporfin was dissolved in phosphate-buffered saline containing 10% DMSO and 0 - 100 mg/kg was delivered by intraperitoneal injection of 100 μl three times per week (M/W/F). Five mice were used per group (two tumors per mouse) and treatment was initiated two days after tumor cell injection. Tumor growth was monitored by measuring tumor diameter and calculating tumor volume using the formula, volume = 4/3π x (diameter/2)^3^. Mice were euthanized by injection of 250 μl of a 2.5% stock of Avertin per mouse followed by cervical dislocation of the neck. Tumor samples were harvested to prepare extract for immunoblot and sections for immunostaining. These experiments were reviewed and approved by the University of Maryland-Baltimore Institutional Animal Care and Use Committee. The plotted values are mean ± SEM and significance was determined using the students t-test.

### Matrigel invasion of tumor-derived cells

Tumors were initiated and treated with PLX4032 or verteporfin as above. At 4 wk the tumors were removed, mechanically dissociated and dispersed as single cell suspensions with 0.25% trypsin for 10 min and plated as monolayer cultures. After 24 h, the cells were harvested and seeded at 25,000 cells/well atop a 0.1 ml matrigel layer in Millicell (1 cm diameter, 8 μm pore size) chambers in the presence of a serum gradient in the absence of drug treatment [38]. After 18 h, the membranes were stained with DAPI and the nuclei of migrated cells were visualized by inverted fluorescence microscopy [38].

RETRACTED

### qRT-PCR analysis of mRNA level

Total RNA was isolated using Illustra RNAspin mini kit (GE Healthcare), and 1 μg of RNA was used for cDNA synthesis. Gene expression was measured by real time PCR using Light Cycler 480 SYBR Green I Master Mix (04-707 516 001) from Roche Diagnostics (Indianapolis, IN, USA). The signals were normalized using cyclophilin A control primers. The gene specific primers used for detection of mRNA levels were as follows: cyclophilin A (forward, 5′-CAT CTG CAC TGF CAA GAC TGA; reverse, 5′-TTC ATG CCT TCT TTC ACT TTG C), TAZ (forward, 5′-GTA TCC CAG CCA AAT CTC G; reverse, 5′-TTC TGA GTG GGG TGG TTC) and YAP1 (forward, 5′-GTGAGCCCACAGGAGTTAGC; reverse, 5′-CTCGAGAGTGATAGGTGCCA) [11].
